# Ginsenoside Rg1 Ameliorates Acute Renal Ischemia/Reperfusion Injury via Upregulating AMPK*α*1 Expression

**DOI:** 10.1155/2022/3737137

**Published:** 2022-09-01

**Authors:** Qing Zhou, Xinlan He, Xiaoyu Zhao, Qigui Fan, Songqing Lai, Dan Liu, Huan He, Ming He

**Affiliations:** ^1^Institute of Cardiovascular Diseases, Jiangxi Academy of Clinical Medical Sciences, The First Affiliated Hospital of Nanchang University, Nanchang 330006, China; ^2^Jiangxi Provincial Key Laboratory of Basic Pharmacology, Nanchang University School of Pharmaceutical Science, Nanchang 330006, China

## Abstract

Acute renal ischemia/reperfusion (I/R) injury often occurs during kidney transplantation and other kidney surgeries, and the molecular mechanism involves oxidative stress. We hypothesized that ginsenoside Rg1 (Rg1), a saponin derived from ginseng, would protect the renal tissue against acute renal I/R injury by upregulating 5′ adenosine monophosphate-activated protein kinase *α*1 (AMPK*α*1) expression and inhibiting oxidative stress. The models of acute anoxia/reoxygenation (A/R) damage in normal rat kidney epithelial cell lines (NRK-52E) and acute renal I/R injury in mice were constructed. The results revealed that pretreatment with 25 *μ*M Rg1 significantly increased NRK-52E viability, decreased lactate dehydrogenase (LDH) activity and apoptosis, suppressed reactive oxygen species generation and oxidative stress, stabilized mitochondrial membrane potential and reduced mitochondria permeability transition pore openness, decreased adenosine monophosphate/adenosine triphosphate ratio, and upregulated the expression of AMPK*α*1, cytochrome b-c1 complex subunit 2, NADH dehydrogenase (ubiquinone) 1 beta subcomplex subunit 8, and B-cell lymphoma 2, while downregulating BCL2-associated X protein expression. The effects of Rg1 pretreatment were similar to those of pAD/Flag-AMPK*α*1. After acute renal I/R injury, serum creatinine, blood urea nitrogen, LDH activity, and oxidative stress in renal tissue significantly increased. Rg1 pretreatment upregulated AMPK*α*1 expression, which protects against acute renal I/R injury by maintaining renal function homeostasis, inhibiting oxidative stress, and reducing apoptosis. Compound C, a specific inhibitor of AMPK, reversed the effects of Rg1. In summary, Rg1 pretreatment upregulated AMPK*α*1 expression, inhibited oxidative stress, maintained mitochondrial function, improved energy metabolism, reduced apoptosis, and ultimately protected renal tissue against acute renal I/R injury.

## 1. Introduction

Acute renal injury (AKI) is a prevalent pathophysiological condition [1]. Ischemic injury is one of the most common AKI due to abundant renal blood flow. Recovering blood flow is the most effective treatment, but blood reperfusion causes inevitable damage. This process is called renal ischemia/reperfusion (I/R) injury. Acute renal I/R injury is divided into two stages. First, a lack of oxygen and nutrient supply during the ischemia phase induces kidney damage. However, during the reperfusion phase, intracellular reactive oxygen species (ROS) are generated, and the intracellular redox balance is disrupted, resulting in more severe renal injury than during the ischemic period. Therefore, reperfusion injury is dominated by excessive oxidative stress [2, 3]. Some researchers have studied the activities of enzymes and levels of nonenzymatic components involved in the antioxidant defense. The study concluded that acute renal I/R damage caused by renal transplantation might partly depend on the extent of oxidative stress [3].

Ginsenoside Rg1 (Rg1), a phytochemical, is one of the active ingredients in ginseng, a traditional Chinese medicine. Rg1 has antioxidant activity that reduces ROS generation. The characteristic of antioxidant stress in Rg1 is intimately related to its neuroprotective effect [4]. Rg1 mitigates excessive ROS generation induced by dopamine, restrains the release of mitochondrial cytochrome C (Cyt C), and declines oxidative stress [5]. Rg1 also reduces cardiac oxidative stress, which may be mediated by the AMPK/Nrf2/HO-1 pathway [6]. The combination of Rg1 and intravenous astragaloside weakens diabetic nephropathy by abating oxidative stress [7]. There are few reports about the protective effect of Rg1 on the ischemic kidney [8].

5′ adenosine monophosphate-activated protein kinase (AMPK), a heterotrimer, is an intracellular energy sensor. When cells suffer stress, such as energy deprivation and oxidative stress, AMPK detects changes in adenosine monophosphate (AMP) or adenosine triphosphate (ATP). AMPK is activated to promote ATP production and reduce ATP consumption, thereby maintaining energy balance and resisting external stimulation [9]. Previous studies have confirmed the importance of AMPK-mediated mitophagy in alleviating oxidative stress [10]. Persistent mitochondrial dysfunction is a significant factor in the early progression of kidney diseases, such as AKI and diabetic nephropathy, because of the renal function [11]. Mitochondrial dysfunction also induces ATP production reduction, cell dysfunction, structural changes, and renal function loss [12]. Therefore, the homeostasis of mitochondrial function is essential for normal renal function [11]. AMPK, as a gatekeeper of metabolism and mitochondrial homeostasis, has gained wide attention [9, 12] as a potential therapeutic target for many diseases [13]. Rg1 exerts various cytoprotection by activating AMPK expression, including influencing glucose uptake in insulin-resistant muscle cells [14], improving nutritional stress injury in H9c2 cells [15], and regulating the autophagy in NRK-52E cells by activating the AMPK/mTOR pathway [16].

Therefore, this study was aimed at investigating *in vivo* and *in vitro* (1) whether Rg1 pretreatment protected renal tissue against acute I/R injury, (2) whether Rg1 pretreatment exerted renal protection by upregulating AMPK*α*1 expression, and (3) whether Rg1 pretreatment inhibited oxidative stress, improved mitochondrial function, and alleviated apoptosis by upregulating AMPK*α*1 expression against acute renal I/R injury.

## 2. Materials and Methods

### 2.1. Materials, Cells, and Animals

Adenovirus pAD/Flag-AMPK*α*1 was purchased from GeneChem Co., Ltd. (Shanghai, China). Rg1 (purity ≥ 98%) was purchased from Solarbio (cat. no. SG8330, Shanghai, China). Compound C was acquired from Selleck (Houston, USA). Antibodies directed against AMPK*α*1, cytochrome b-c1 complex subunit 2 (UQCRC2), NADH dehydrogenase (ubiquinone) 1 beta subcomplex subunit 8 (NDUFB8), and Cyt C were obtained from Abcam (Cambridge, UK). Antibodies directed against Bax, Bcl-2, cleaved caspase 3, cytochrome c oxidase subunit IV (COXIV), and glyceraldehyde-3-phosphate dehydrogenase (GAPDH) were obtained from Cell Signaling Technology (Boston, USA). A horseradish peroxidase-conjugated IgG secondary antibody was purchased from Zsbio (Beijing, China).

The normal rat kidney epithelial cell line (NRK-52E) was acquired from the Chinese infrastructure of cell line resources (Shanghai, China). Adult male C57BL/6 mice (8 weeks old, weighing about 20 g) were furnished by the animal center of Nanchang University (Nanchang, China). All experimental procedures followed the National Institutes of Health (NIH) Guidelines for the Care and Use of Laboratory Animals (NIH Publication No. 85-23, revised 1996) and were approved by the Ethics Committee of Nanchang University (no. 2021-0026).

### 2.2. In Vitro Experiments

#### 2.2.1. Cell Culture and Acute Anoxia/Reoxygenation (A/R) Damage Model

NRK-52E cells were cultured in Dulbecco's modified Eagle's medium (DMEM), which contained 4.5 g/L glucose supplemented with 5% fetal bovine serum (FBS, Solarbio, Shanghai, China), penicillin (100 IU/mL), and streptomycin (100 mg/mL) in a humidified incubator with 5% carbon dioxide (CO_2_) in a 37°C atmosphere.

The acute A/R damage model of NRK-52E cells was induced by 4 h anoxia and 12 h reoxygenation. In the anoxia stage, the cells were fostered for 4 h under anoxia conditions (95% nitrogen (N_2_) and 5% CO_2_) in a medium without nutrients. In reoxygenation, the cells above were transferred into a serum-free medium and returned to a standard incubator (5% CO_2_ and 95% air) for 12 h [17, 18].

#### 2.2.2. In Vitro Experiment Design

The experimental design used in this study was as follows: (1) the control group: NRK-52E cells were cultured under normal conditions; (2) the A/R group: NRK-52E cells were exposed to 4 h anoxia and 12 h reoxygenation; (3) the Rg1+A/R group: the acute A/R injury model of NRK-52E cells was established after the cells were handled with 25 *μ*M Rg1 for 24 h; (4) the pAD/Flag-AMPK*α*1+A/R group: pAD/Flag-AMPK*α*1 was added to NRK-52E cells for 24 h before acute A/R injury; and (5) the compound C+Rg1+A/R group: similar treatment was performed with the Rg1+A/R group, and only 5 *μ*M compound C [19] was added 2 h before 25 *μ*M Rg1 treatment.

#### 2.2.3. Cell Counting Kit (CCK-8) and Lactate Dehydrogenase (LDH) Activity Assay

Cells were seeded in 96-well plates with 1 × 10^4^ cells/well. Following cell treatment, the culture supernatant was discarded. Ten microliters of CCK-8 (5 mg/mL) reagents was mixed with 100 *μ*L of DMEM medium, and the mixture was used for detecting cell viability at a 37°C incubator for 2–3 h. A spectrophotometer was used to measure absorbance at 450 nm (Bio-Rad680). The cell viability was presented as percentage relative to the control group.

LDH is an intracellular enzyme that is released when the cell membrane ruptures [20]. Therefore, LDH activity in the culture supernatant was detected after cells were treated according kit instructions (Jiancheng, Nanjing, China).

#### 2.2.4. Assessment of Oxidative Stress

When cells and tissues are exposed to anoxia or other stresses, the endogenous antioxidant enzyme system is activated. The status of this system can be reflected by catalase (CAT), glutathione peroxidase (GSH-Px), and superoxide dismutase (SOD) activity [21]. The malondialdehyde (MDA) content, one of the most widely accepted lipid peroxidation biomarkers, is also used for indicating oxidative stress [22]. At the time of detection, NRK-52E cells or renal tissue homogenates were prepared, and the activities of CAT, GSH-Px and SOD, and MDA content were determined according to the instructions (Jiancheng, Nanjing, China), respectively.

The CAT activity was measured at 405 nm and calculated by the following formula:

(1) $$\begin{array}{c} CAT\;activity\;\left(U/mg\;prot\right)=\left(\frac{\left({Control}_{OD}-{Determination}_{OD}\right)\times 271\times \left[1/\left(60\times sampling\;volume\right)\right]}{sample\;protein\;concentration}\right). \end{array}$$

The GSH-Px activity was detected at 412 nm and calculated by the following formula:

(2) $$\begin{array}{c} GSH‐Px\;activity\;\left(U/g\;prot\right)=\frac{\left(nonenzyme\;{tube}_{OD}-enzyme\;{tube}_{OD}\right)/\left(standard\;{tube}_{OD}-blank\;{tube}_{OD}\right)\times 20\times 5}{reaction\;time/\left(sampling\;volume\times sample\;protein\;concentration\right)}. \end{array}$$

The SOD activity was detected at 450 nm and calculated by the following formula:

(3) $$\begin{array}{c} SOD\;inhibition\;rate\;\left(\%\right)=\frac{\left[\left(A_{control}-A_{control\;blank}\right)-\left(A_{determination}-A_{control\;blank}\right)\right]}{A_{control}-A_{control\;blank}},\\ SOD\;activity\;\left(U/mg\;prot\right)=\frac{SOD\;inhibition\;rate/50\%\times \left(reaction\;system/dilution\;multiple\right)}{sample\;protein\;concentration\;\left(mg/ml\right)}. \end{array}$$

The MDA content was detected at 532 nm and calculated by the following formula:

(4) $$\begin{array}{c} MDA\;content\;\left(nmol/mg\;prot\right)=\frac{\left({determination}_{OD}-{Blank}_{OD}\right)/\left({standard}_{OD}-{Blank}_{OD}\right)\times Standard\;\left.concentration\right)}{sample\;protein\;concentration}. \end{array}$$

Reduced glutathione, an essential antioxidant, is crucial in maintaining the redox state of protein sulfhydryl groups [23, 24]. The reduced glutathione (GSH) and oxidized glutathione (GSSG) levels of NRK-52E's lysed supernatants were measured following the manufacturer's instructions (Beyotime, Haimen, China). Total glutathione and GSSG were detected at 412 nm, and

(5) $$\begin{array}{c} GSH=total\;glutathione-GSSG\times 2. \end{array}$$

Subsequently, the GSH/GSSG ratio was calculated.

As previously reported, intracellular ROS generation was detected with a 6-carboxy-2′-7′-dichlorodihydro-fluorescein diacetate (DCFH-DA) probe (Thermo Fisher Scientific, USA) by flow cytometry analysis (Cytomics FC500, Ex = 488 nm, Em = 525 nm, Beckman Coulter, Brea, CA, USA) [25].

#### 2.2.5. Assessment of Mitochondrial Membrane Potential (MMP)

The MMP loss of NRK-52E cells stained with 5,5′,6,6′-tetrachloro-1,11′,3,3′-tetraethyl-benzimidazole carbocyanine iodide (JC-1) probe (BestBio, Shanghai, China) was assessed by flow cytometry (Cytomics FC500, Ex = 488 nm, Em = 530 nm). The loss of MMP was presented by the ratio of red to green fluorescence intensity (the ratio of fluorescence in the upper right quadrant and lower right quadrant) [26].

#### 2.2.6. Assessment of Mitochondrial Permeability Transition Pore (mPTP) Openness

mPTP is a protein complex that exists between the mitochondria's inner and outer membrane, which plays an essential role in cell survival and apoptosis. As previously reported, the mitochondrial swelling assay was used to detect mPTP openness [27]. The mitochondria were separated strictly following the instruction of the mitochondrial isolation kit. The swelling buffer (KCl 120 mM, Tris-HCl 10 mM, MOPS 20 mM, and KH_2_PO_4_ 5 mM) was used to suspend mitochondria, and then, calcium chloride solution was added to stimulate mPTP opening. The mitochondrial density declined at a steady speed. Therefore, the absorbance change at 520 nm every minute indicated the degree of mPTP openness.

#### 2.2.7. Assay of the Intracellular AMP/ATP Ratio

Cells were scraped, and the homogenate was prepared with phosphate-buffered saline (PBS). The supernatant of the homogenate was acquired after centrifugation at 3000 rpm for 10 min. The AMP, ATP, and AMP/ATP ratios were determined according to the manual of the enzyme-linked immunosorbent assay (ELISA) assay kit [28]. The absorbance of reactants was measured with a microplate at 450 nm.

#### 2.2.8. Determination of Apoptosis

After the corresponding treatment, NRK-52E cells in each group were collected. 5 *μ*L Annexin V-FIFC was added to the cells and incubated in the dark for 15 min. Subsequently, 10 *μ*L propidium iodide (PI) was added and incubated in darkness for 5 min. Finally, the cells were resuspended in PBS, and the apoptosis cells (%) were detected by flow cytometry [29].

DeadEnd™ colorimetric terminal deoxynucleotidyl transferase dUTP nick-end labeling (TUNEL) system (Promega, Wisconsin, USA) was used to evaluate cell apoptosis. At the time of detection, NRK-52E cells were fixed with 4% paraformaldehyde. After permeabilization with 0.2% Triton X-100, NRK-52E cells were incubated in terminal deoxynucleotidyl transferase recombinant (rTdT) reaction mix for 60 min and then incubated with horseradish peroxidase (HRP) solution for 30 min. A solution of 3,3′-diaminobenzidine (DAB) was added for color reaction, and the nucleus was stained with hematoxylin. In *in vivo* experiment, renal tissue was fixed with paraformaldehyde, dehydrated gradiently, embedded, and cut into sections. The sections were incubated and stained with rTdT mix buffer and DAB buffer, respectively. The nucleus was stained with hematoxylin and was visualized under the microscope (Olympus, Tokyo, Japan). TUNEL-positive (apoptosis) spots are brown, while the nucleus is blue [30]. TUNEL-positive spots were presented as a control group fold.

Following the appropriate treatment, NRK-52E cells were harvested, lysed, and centrifuged to obtain the supernatant. The supernatant of each group with the same protein concentration was used to detect caspase 3 activity. The reaction system was established according to the instructions for determining caspase 3 activity at 405 nm [31]. The relative caspase 3 activity of each group was expressed as experimental group_OD_/control group_OD_.

#### 2.2.9. Western Blot Analysis

Following the appropriate treatment, NRK-52E cells and renal tissue samples were extracted using a protein extraction kit (Applygen Technologies, Beijing, China). The protein content was measured by a bicinchoninic acid (BCA) protein assay kit (Thermo Fisher, USA). Thirty micrograms of protein were loaded and separated on 12% sodium dodecyl sulfate-polyacrylamide gel electrophoresis (SDS-PAGE) and transferred to polyvinylidene fluoride membranes. The membranes were blocked with 5% milk and incubated at 4°C overnight in primary antibodies (AMPK*α*1, 1 : 500; UQCRC2, 1 : 1000; NDUFB8, 1 : 1000; Cyt C, 1 : 1000; COXIV, 1 : 1000; cleaved caspase-3, 1 : 500; Bax, 1 : 1000; Bcl-2, 1 : 1000; and GAPDH, 1 : 1000). Subsequently, the primary antibodies were removed, and the HRP-conjugated secondary antibodies were blotted for 2 h. Finally, the protein bands were observed by Image Lab Software (Bio-Rad, USA).

### 2.3. In Vivo Experiments

#### 2.3.1. Acute Renal I/R Injury Model

C57BL/6 mice were fed conventionally (23 ± 2°C, humidity: 50% ± 5%, a 12 h light/dark cycle). After 24 h of experimental treatment, mice were anesthetized with ketamine (100 mg/kg) and xylazine (8 mg/kg) intraperitoneally. The abdominal cavity was opened, and the bilateral renal pedicle was clamped by noninvasive arterial clamps. The kidneys went from pink to dark red within 5 min. The arterial clamps were removed after 30 min, and the kidneys returned to pink within 5 min, indicating the successful establishment of renal I/R injury. Finally, the abdominal cavity was sutured and reperfused for 24 h [32].

#### 2.3.2. In Vivo Experiment Grouping

In this study, 24 mice were randomly divided into four groups: (1) the sham group: mice were exposed to sham operation; (2) the I/R group: mice suffered acute renal I/R injury; (3) the Rg1+AR group: mice were treated with 40 mg/kg Rg1 [33] intraperitoneally once a day for 2 weeks before acute renal I/R injury; and (4) the compound C+Rg1+I/R group: similar to the Rg1+AR group, only 5 mg/kg compound C [34] was administrated intraperitoneally 2 h before Rg1 treatment.

#### 2.3.3. Evaluation of Serum LDH Activity, Serum Creatinine (Scr) Levels, and Blood Urea Nitrogen (BUN)

After 24 h of reperfusion, the mice were routinely anesthetized. The blood of the mice was collected and centrifuged at 4°C and 3000 rpm for 10 min, and the serum was obtained. The reaction system was established according to the instructions, and the absorbance was detected with a spectrophotometer. The LDH activity, Scr levels, and BUN were directly proportional to the absorbance.

#### 2.3.4. Hematoxylin and Eosin (H&E) Staining

After the appropriate treatment, kidneys were routinely dehydrated, embedded, and sliced. Kidney tissue sections were subjected to gradient ethanol hydration. Subsequently, kidney tissue sections were stained with hematoxylin for 5 min and eosin for 1 min. Finally, kidney tissue sections were dehydrated with gradient alcohol, sealed with neutral gum, and examined microscopically.

### 2.4. Statistical Analysis

Data are presented as the mean ± standard deviation (SD). One-way analysis of variance was employed to test the significance of differences in the biochemical data across groups, followed by post hoc Tukey's honestly significant difference testing for individual differences. Differences with *p* < 0.05 were considered significant.

## 3. Results

### 3.1. Rg1 Pretreatment Ameliorated Acute A/R Damage in NRK-52E Cells

To explore whether the phytochemical, Rg1, has a protective effect on acute A/R damage in NRK-52E cells, we measured cell viability and LDH activity, respectively. The increased LDH activity and decreased cell viability in the A/R group (*p* < 0.01) revealed that the acute A/R model was successfully established (Figures 1(a) and 1(b)). Rg1 pretreatment protected NRK-52E cells against acute A/R injury in a concentration-dependent manner (*p* < 0.05). Therefore, 25 *μ*M Rg1 was used in the following experiments.

Compared to the A/R group, 25 *μ*M Rg1 pretreatment had similar effects on pAD/Flag-AMPK*α*1, which increased NRK-52E cell viability and decreased LDH activity (Figures 1(c) and 1(d), *p* < 0.01), indicating that Rg1 pretreatment effectively protected NRK-52E cells against acute A/R injury by increasing AMPK*α*1 expression.

### 3.2. Rg1 Pretreatment Rescued Oxidative Stress-Induced Acute A/R Damage in NRK-52E Cells

To identify the role of oxidative stress in acute A/R injury in NRK-52E cells, the oxidative stress biomarkers and activities of CAT, SOD, and GSH-Px and MDA levels were detected. Our results revealed that oxidative stress increased after acute A/R damage in NRK-52E cells, which was indicated by the increased MDA concentration and abated activities of CAT, SOD, and GSH-Px (Figures 2(a)–2(d), *p* < 0.01). Thus, we further investigated intracellular ROS generation and GSH/GSSG ratio. The intracellular ROS generation was increased in the A/R group (Figures 2(e) and 2(f), *p* < 0.01). Contrarily, the GSH/GSSG ratio was significantly lower in the A/R group (Figure 2(g), *p* < 0.01), revealing the typical oxidative stress features.

Notably, the above effects were abolished by treating NRK-52E cells with pAD/Flag-AMPK*α*1, and Rg1 pretreatment had similar effects (*p* < 0.01). However, the specific AMPK inhibitor (5 *μ*M compound C) inhibited the effects of Rg1 against oxidative stress in NRK-52E cells (Figure 2(g), *p* < 0.01). All these data suggested that Rg1 exerted antioxidative stress by upregulating AMPK*α*1 expression.

Therefore, these data supported that acute A/R injury induced oxidative stress in NRK-52E cells. The acute A/R injury was improved following pAD/Flag-AMPK*α*1 treatment. Rg1 pretreatment exhibited antioxidative stress effects, possibly by upregulating AMPK*α*1 expression.

### 3.3. Rg1 Pretreatment Protected NRK-52E Cells against Acute A/R Injury by Preserving Mitochondrial Function

Growing evidence indicates that mitochondrial function is impaired after acute A/R injury. MMP serves as a mitochondrial function marker, and MMP loss suggests abnormal mitochondrial function [35]. Figures 3(a) and 3(b) depict the significant MMP loss in the A/R group. The effect of acute A/R injury was significantly reversed after pretreating NRK-52E cells with pAD/Flag- AMPK*α*1 or Rg1 (*p* < 0.01).

On the other hand, another index of mitochondrial function, mPTP openness [36], was detected in the study. Based on our data (Figures 3(c) and 3(d)), mPTP openness was higher in the A/R group (*p* < 0.01). Similarly, the mPTP openness was attenuated apparently after pAD/Flag-AMPK*α*1 or Rg1 pretreatment (*p* < 0.01).

### 3.4. Rg1 Pretreatment Improved Energy Metabolism of NRK-52E Cells after Acute A/R Injury

To confirm the effect of Rg1 on regulating AMPK*α*1 expression, we detected AMPK*α*1 expression in NRK-52E cells. As expected, Rg1 pretreatment significantly upregulated AMPK*α*1 expression (*p* < 0.01, Figures 4(a) and 4(d)).

The mitochondrial respiratory electron transport chain is important in ensuring cell energy supply, and the complex I subunit (NDUFB8) and complex III subunit (UQCRC2) are sensitive to acute A/R injury [37]. Our results demonstrated that NDUFB8 and UQCRC2 expression decreased following acute A/R injury. However, pretreatment with 25 *μ*M Rg1 significantly increased NDUFB8 and UQCRC2 expression. However, 5 *μ*M compound C significantly inhibited NDUFB8 and UQCRC2 expression (*p* < 0.01, Figures 4(a)–4(c)).

The A/R group had a higher AMP/ATP ratio than the control group (Figure 4(e), *p* < 0.01). AMPK, the energy sensor, is activated when there is low ATP generation and high ATP consumption. When there is an increase in energy stress, the AMP/ATP ratio increases [38]. Therefore, compared with the control group, the A/R group had slightly upregulated AMPK*α*1 expression, while Rg1 further upregulated AMPK*α*1 expression, promoted ATP production, and reduced the AMP/ATP ratio. Adding compound C inhibited the expression of AMPK*α*1; thus, improved energy metabolism effect by Rg1 was reversed. Therefore, Rg1 improved energy metabolism by upregulating AMPK*α*1 expression.

### 3.5. Rg1 Restrained Apoptosis Induced by Acute A/R Injury in NRK-52E Cells

Acute A/R injury induced cell apoptosis. Rg1 pretreatment decreased the expression of the proapoptotic protein Bax and increased the expression of the antiapoptotic protein Bcl-2 (Figures 5(a)–5(c), *p* < 0.01).

When mitochondrial function is impaired, Cyt C is released from the mitochondria into the cytosol, activating caspases and ultimately triggering apoptosis [39]. Rg1 pretreatment significantly reduced the translocation of Cyt C from mitochondria to the cytosol, decreased cleaved caspase 3 expressions, and inhibited caspase 3 activity (Figures 5(a) and 5(d)–5(g), *p* < 0.01). The Annexin V-FITC/PI and TUNEL assay revealed that the A/R group exhibited more apparent apoptosis (Annexin V-FITC/PI staining dot plots and TUNEL-positive spots) (Figures 5(h)–5(k)), and Rg1 pretreatment significantly decreased Annexin V-FITC/PI staining dot plots and TUNEL-positive spots. As shown in Figures 5(h)–5(k), Rg1 pretreatment inhibited NRK-52E apoptosis induced by acute A/R injury (*p* < 0.01).

Notably, the above protective effects of Rg1 were abolished with compound C (*p* < 0.05). These data suggest that Rg1 inhibits apoptosis by upregulating AMPK expression.

### 3.6. Rg1 Resumed Acute Renal I/R Injury

The abnormal elevation of Scr and BUN usually indicates renal dysfunction [40], and the increased serum LDH activity indicates cell damage [39]. The I/R group had elevated serum LDH activity and Scr and BUN contents, which deteriorated renal morphology (renal tubular swelling and tubular epithelial cell exfoliation) (Figures 6(a)–6(d), *p* < 0.01). Rg1 pretreatment ameliorated these indexes after acute renal I/R injury. However, compound C reversed the protective effects of Rg1 pretreatment (*p* < 0.01).

### 3.7. Rg1 Alleviated Oxidative Stress Induced by Acute Renal I/R Injury

Oxidative stress is an oxidation and antioxidation disorder that contributes to various diseases [41–43]. We aimed to reconfirm whether oxidative stress leads to acute renal I/R injury. As expected, excess oxidative stress was discovered in the renal I/R group, evidenced by prominently mitigated antioxidant enzyme activities such as CAT, SOD, and GSH-Px and abnormally accumulated lipid peroxidation products of MDA (Figures 7(a)–7(d), *p* < 0.01). Similar to *in vitro*, the excellent antioxidant stress effects of Rg1 pretreatment were inhibited by compound C (*p* < 0.01).

### 3.8. Rg1 Mitigated Apoptosis Induced by Acute Renal I/R Injury

We detected the apoptosis-related indexes to confirm the relationship between acute renal I/R injury and apoptosis. As shown in Figures 8(a) and 8(b), Rg1 significantly reduced the TUNEL-positive spots (*p* < 0.05). The expression of apoptosis-related proteins (Bax and cleaved caspase 3) was inhibited, and Bcl-2 and AMPK*α*1 expression was increased by Rg1 pretreatment (Figures 8(c)–8(g), *p* < 0.01). On the contrary, compound C and Rg1 cotreatment did not protect against acute renal I/R damage (*p* < 0.05). These results indicated that the antiapoptotic effect of Rg1 was related to the upregulation of AMPK*α*1 expression.

## 4. Discussion

The kidney is a vital excretory organ with a distinct tubular structure. Renal perfusion is abundant, and renal blood flow accounts for 25% of cardiac output, which is sensitive to ischemia (anoxia) [44]. When the kidney is continuously ischemic, the capillaries loosen, and the renal tubules are damaged; the secretion of vascular endothelial growth factor by renal tubular epithelial cells is reduced, which further aggravates ischemia and forms a vicious circle [45]. The reperfusion (reoxygenation) process causes more severe damage. Acute renal I/R injury is generally caused by acute renal blood flow reduction and insufficient supply of oxygen and nutrition because of renal transplant, massive bleeding, contrast media, trauma, sepsis, or major surgeries. Common symptoms are the rapid increase in creatinine, oliguria, or no urine. Therefore, it is urgent to clarify the mechanism of acute renal I/R injury and reduce clinical complications. Our study focused on the relationship between oxidative stress and acute renal I/R injury.

Oxidative stress is an imbalance state between oxidation and antioxidation. It has been reported that oxidative stress is closely related to many diseases. Moreover, the relationship between oxidative stress and acute renal I/R injury has been reported [46], which has also been verified *in vivo* and *in vitro* in this study (Figures 2 and 6). However, we aimed to find the antioxidative stress drugs, especially natural phytochemicals, to provide new ideas for treating related diseases.

Phytochemicals have attracted extensive attention because of their multitarget, multimechanism, and multimedicinal values [47, 48]. Rg1, a saponin phytochemical isolated from ginseng, has been studied as a major active ingredient to expand knowledge background and application prospects. Whether Rg1 has protective effects against acute renal I/R injury and the specific mechanism are still unclear. Compared with salvage treatment after acute renal I/R injury, pharmacological preconditioning, especially nutritional preconditioning, is essential against acute renal I/R injury. Hence, our study explored the protective effects of Rg1 pretreatment against acute renal I/R injury *in vivo* and *in vitro*. Our study revealed that Rg1 pretreatment simulated by pAD/Flag-AMPK*α*1 protected NRK-52E cells against acute A/R injury, increased NRK-52E cell viability, activities of endogenous antioxidant enzymes, and GSH/GSSG ratio, decreased LDH activity and MDA content, and inhibited ROS generation (Figures 1 and 2). Rg1 pretreatment significantly improved renal dysfunction caused by acute renal I/R injury *in vivo* (Figure 6). After acute renal I/R injury, the strengthened oxidative stress was significantly inhibited by Rg1 pretreatment (Figure 7). It should be noted that the renal protection and oxidative stress inhibition of Rg1 pretreatment *in vivo* and *in vitro* were achieved by upregulating AMPK*α*1 expression (Figures 4(a) and 8(b)). However, these effects were significantly weakened by compound C. This view is consistent with the SIRT1/AMPK pathway, which inhibits ROS generation [45].

The kidney requires energy to remove various wastes from the blood. The content of renal mitochondria is second only to the heart. Mitochondrial functional homeostasis is the basis of healthy renal function. The structural integrity of the mitochondrial membrane is essential for mitochondrial function. MMP loss and mPTP openness lead to mitochondrial Cyt C release into the cytosol and activate the caspase pathway, triggering apoptosis. After acute renal I/R injury, mitochondrial morphology, function, and related pathways were changed, leading to renal injury [11]. Fortunately, the process is reversible. AMPK is a heterotrimer composed of *α*, *β*, and *γ* subunits. Activation of AMPK promotes ATP production and reduces ATP consumption to maintain energy homeostasis. AMPK*α*1, as the main subunit in the kidney, has attracted our attention. In this study, Rg1 pretreatment or pAD/Flag- AMPK*α*1 stabilized MMP and reduced mPTP openness and mitochondrial Cyt C release to the cytosol (Figures 3–5). These results are consistent with previous reports [49]. More importantly, Rg1 pretreatment promoted mitochondrial respiratory chain complex NDUFB8 and UQCRC2 expression and ATP production. These data reveal that mitochondrial energy metabolism was improved. Similarly, Rg1 pretreatment maintained mitochondrial function and improved energy metabolism by upregulating AMPK*α*1 expression (Figure 4(a)).

Excessive oxidative stress caused by acute A/R and I/R injury induces mitochondrial dysfunction and energy metabolism disorder, leading to apoptosis. In this study, the renal tissue and NRK-52E cells had apoptosis *in vitro* and *in vivo* after the related injury, which was confirmed by the related protein expressions, as well as Annexin V-FITC/PI staining dot plots, TUNEL-positive spots, and caspase 3 activity. Rg1 pretreatment effectively alleviated apoptosis by upregulating AMPK*α*1 expression (Figures 5 and 8).

## 5. Conclusion

In summary, oxidative stress induced by acute renal I/R injury caused excessive intracellular ROS generation and lipid peroxidation accumulation, inhibited the activities of endogenous antioxidative enzymes, damaged mitochondrial function and suppressed energy metabolism, and ultimately induced renal apoptosis. Rg1 pretreatment upregulated AMPK*α*1 expression, inhibited oxidative stress, maintained mitochondrial function, improved energy metabolism, reduced renal apoptosis, and protected renal tissue against acute I/R injury, mimicking the effects of pAD/Flag-AMPK*α*1, and the effects were weakened by compound C.

## Figures and Tables

**Figure 1:** Rg1 pretreatment protected NRK-52E cells against acute A/R injury. NRK-52E cells suffered 4 h anoxia and 12 h reoxygenation to induce acute A/R damage. Rg1 pretreatment increased cell viability and decreased LDH activity in a concentration-dependent manner. (a, c) Cell viability (%) detected by CCK-8. (b, d) LDH activity released into the culture media. Data are expressed as mean ± SD for three individual experiments. ^a^*p* < 0.01 vs. the control group. ^b^*p* < 0.01 vs. the A/R group.

**Figure 2:** Rg1 pretreatment ameliorated oxidative stress caused by acute A/R injury in NRK-52E cells. (a) MDA content. (b) CAT activity. (c) GSH-Px activity. (d) SOD activity. (e) Intracellular ROS generation was measured by flow cytometry. (f) Histogram of the intracellular ROS generation. (g) Histogram of the GSH/GSSG ratio. Data are presented as the mean ± SD for 3 individual experiments. ^a^*p* < 0.01 vs. the control group. ^b^*p* < 0.01 vs. the A/R group. ^c^*p* < 0.01 vs. the Rg1+A/R group.

**Figure 3:** Rg1 pretreatment stabilized mitochondrial function after acute A/R injury. (a) Mitochondrial membrane potential (MMP) level was determined by flow cytometry (red dots represent cells, and the cells moved from up to down, indicating MMP loss). (b) Histogram of the red or green fluorescence ratio (the ratio of fluorescence density in the upper right quadrant and lower right quadrant). (c) Mitochondrial permeability transition pore (mPTP) openness is shown by the degree of decrease in absorbance. (d) Histogram of mPTP openness. Data are presented as mean ± SD for three individual experiments. ^a^*p* < 0.01 vs. the control group. ^b^*p* < 0.01 vs. the A/R group.

**Figure 4:** Rg1 pretreatment promoted energy metabolism of NRK-52E cells after acute A/R injury. (a) The expression of NDUFB8, UQCRC2, and AMPK*α*1 in NRK-52E cells. (b) Histogram of NDUFB8 expression. (c) Histogram of UQCRC2 expression. (d) Histogram of AMPK*α*1 expression. (e) Histogram of the AMP/ATP ratio measured by ELISA. Data are presented as the mean ± SD for three individual experiments. ^a^*p* < 0.01 vs. the control group. ^b^*p* < 0.01 vs. the A/R group. ^c^*p* < 0.01 vs. the Rg1+A/R group.

**Figure 5:** Rg1 pretreatment mitigated apoptosis induced by acute A/R injury. (a) The expression of Bcl-2, Bax, and cleaved caspase 3 in NRK-52E cells. (b) Histogram of cleaved caspase 3 expression. (c) Histogram of Bax expression. (d) Histogram of Bcl-2 expression. (e) Cyt C expression in the cytosol and histogram of Cyt C expression. (f) Cyt C expression in the mitochondria and histogram of Cyt C expression. (g) Histogram of caspase 3 activity. (h) NRK-52E cell apoptosis was analyzed by flow cytometry. (i) Histogram of apoptosis cells (%). (j) TUNEL kits detected cell apoptosis; red arrows indicate TUNEL-positive spots. Scale bars: 50 *μ*m. (k) Histogram of TUNEL-positive spots (fold of control). Data are presented as the mean ± SD for three individual experiments. ^a^*p* < 0.01 vs. the control group. ^b^*p* < 0.01 vs. the A/R group. ^c^*p* < 0.05 vs. the Rg1+A/R group.

**Figure 6:** Rg1 pretreatment improved renal function and morphology after acute renal I/R injury. (a) Histogram of serum LDH activity. (b) Histogram of Scr content. (c) Histogram of BUN content. (d) Representative pictures of H&E staining of kidney sections. Scale bars: 20 *μ*m. After acute renal I/R injury, renal tubular swelling, and tubular epithelial cell exfoliation, Rg1 pretreatment significantly improved renal morphology. Data are presented as the mean ± SD for six individual experiments. ^a^*p* < 0.01 vs. the sham group. ^b^*p* < 0.01 vs. the I/R group. ^c^*p* < 0.01 vs. the Rg1+I/R group.

**Figure 7:** Rg1 pretreatment inhibited oxidative stress induced by acute renal I/R damage. (a) Histogram of MDA content in the renal tissue. (b) Histogram of CAT activity in the renal tissue. (c) Histogram of GSH-Px activity in the renal tissue. (d) Histogram of SOD activity in the renal tissue. Data are presented as the mean ± SD for six individual experiments. ^a^*p* < 0.01 vs. the sham group. ^b^*p* < 0.01 vs. the I/R group. ^c^*p* < 0.01 vs. the Rg1+I/R group.

**Figure 8:** Rg1 pretreatment attenuated the enhanced apoptosis induced by renal I/R damage. (a) TUNEL kits analyzed apoptosis; red arrows indicate TUNEL-positive spots in the renal tissue. Scale bars: 20 *μ*m. (b) Histogram of TUNEL-positive spots (fold of sham). (c) The expression of AMPK*α*1, Bcl-2, Bax, and cleaved caspase 3 in renal tissue. (d) Histogram of cleaved caspase 3 expression. (e) Histogram of Bax expression. (f) Histogram of Bcl-2 expression. (g) Histogram of AMPK*α*1 expression. Data are presented as the mean ± SD for six individual experiments. ^a^*p* < 0.01 vs. the sham group. ^b^*p* < 0.05 vs. the I/R group. ^c^*p* < 0.05 vs. the Rg1+I/R group.

## Data Availability

The data used to support the findings of this study are included within the article.

## Abbreviations

A/R: Anoxia/reoxygenation
ANOVA: Analysis of variance
BUN: Blood urea nitrogen
Cyt C: Cytochrome C
CAT: Catalase
DCFH-DA: 6-Carboxy-2′-7′-dichlorodihydro-flurescein diacetate
DMEM: Dulbecco's modified Eagle's medium
FBS: Fetal bovine serum
GSH: Reduced glutathione
GSH-Px: Glutathione peroxidase
GSSG: Oxidized glutathione
H&E: Hematoxylin and eosin
HRP: Horseradish peroxidase
I/R: Ischemia/reperfusion
JC-1: 5,5′,6,6′-Tetrachloro-1,1′,3,3′-tetraethyl-benzimidazolo carbocyanine iodide
LDH: Lactate dehydrogenase
MDA: Malondialdehyde
MMP: Mitochondrial membrane potential
mPTP: Mitochondrial permeability transition pore
NDUFB8: NADH dehydrogenase (ubiquinone) 1 beta subcomplex subunit 8
NRK-52E: Rat kidney epithelial cell
PBS: Phosphate-buffered saline
Rg1: Ginsenoside Rg1
Rpm: Revolution per minute
ROS: Reactive oxygen species
SD: Standard deviation
SOD: Superoxide dismutase
Scr: Serum creatinine
TUNEL: Terminal deoxynucleotidyl transferase dUTP nick-end labeling
UQCRC2: Cytochrome b-c1 complex subunit 2.
